The article "Therapeutic effect of molecular hydrogen in corneal UVB-induced oxidative stress and corneal photodamage" was retracted in 2021. Reason: duplicated images.

# Therapeutic effect of molecular hydrogen in corneal UVB-induced oxidative stress and corneal photodamage

**DOI:** 10.1038/s41598-017-18334-6

**Published:** 2017-12-21

**Authors:** Cestmir Cejka, Jan Kossl, Barbora Hermankova, Vladimir Holan, Sarka Kubinova, John H. Zhang, Jitka Cejkova

**Affiliations:** 1 Institute of Experimental Medicine of the Czech Academy of Sciences, 14220 Prague 4, Czech Republic; 2 Faculty of Natural Science, Charles University, Vinicna 7, 12843 Prague 2, Czech Republic; 3 Loma Linda University School of Medicine, Loma Linda, CA 92350 USA

## Abstract

The aim of this study is to examine whether molecular hydrogen (H_2_) is able to reduce oxidative stress after corneal damage induced by UVB irradiation. We previously found that UVB irradiation of the cornea caused the imbalance between the antioxidant and prooxidant enzymes in the corneal epithelium, followed by the imbalance between metalloproteinases and their physiological inhibitors (imbalances in favour of prooxidants and metalloproteinases) contributing to oxidative stress and development of the intracorneal inflammation. Here we investigate the effect of H_2_ dissolved in PBS in the concentration 0.5 ppm wt/vol, applied on rabbit corneas during UVB irradiation and healing (UVB doses 1.01 J/cm^2^ once daily for four days). Some irradiated corneas remained untreated or buffer treated. In these corneas the oxidative stress appeared, followed by the excessive inflammation. Malondiladehyde and peroxynitrite expressions were present. The corneas healed with scar formation and neovascularization. In contrast, in H_2_ treated irradiated corneas oxidative stress was suppressed and malondiladehyde and peroxynitrite expressions were absent. The corneas healed with the restoration of transparency. The study provides the first evidence of the role of H_2_ in prevention of oxidative and nitrosative stress in UVB irradiated corneas, which may represent a novel prophylactic approach to corneal photodamage.

## Introduction

UVB (290–320 nm) exposure of the target organs, such as skin or eyes, (particularly the cornea), causes a generation of free radicals and related reactive oxygen species (ROS)^1^. ROS generated as a consequence of UVB radiation, produce oxidative stress in the cornea when the formation of ROS exceeds the antioxidant defence ability of cells. After UVB irradiation, corneal epithelial ROS-generating oxidases contribute to the antioxidant/prooxidant imbalance, in favour of prooxidants, and to the oxidative stress in the cornea^2–7^. The antioxidant/prooxidant enzymatic imbalance is followed by the protease/antiprotease imbalance in the corneal epithelium. We have described the imbalance between matrix metalloproteinases (MMPs) and the tissue inhibitors of metalloproteinases (TIMPs) in favor of MMPs^5,6^. This imbalance contributed to the proinflammatory cytokine induction and to the development of the intracorneal inflammation. Nitric oxide synthases, that generate nitric oxide, were highly expressed in UVB irradiated corneas and the formation of cytotoxic peroxynitrite (NT) (demonstrated by nitrotyrosine residues) in the cornea appeared^8,9^. Corneal hydration and light absorption were increased in untransparent and vascularized corneas. In this study we found that the described disturbances appeared in untreated or PBS treated UVB irradiated corneas, whereas after H_2_ treatment beneficial results in corneal healing were obtained. The UVB induced photodamage was reduced. This is in accordance with previous studies in which H_2_ proved to be effective in the healing of many diseased organs and tissues, in which oxidative stress was involved^10–22^. H_2_ neutralizes the hydroxyl radical and NT inside the cells^10^. Moreover, beside antioxidant activities, H_2_ was shown to exhibit multiple functions, including anti-inflammatory, anti-apoptotic and anti-allergic effects^23,24^. H_2_ regulates various signal transduction pathways and the expression of various genes^16,21^. In ocular diseases and injuries, H_2_ proved neuroprotective and antioxidative effects in acute retinal ischemia reperfusion injury^25,26^ and protective effects against oxidative stress, caused by NT derived from nitric oxide in rat retina^27^. Moreover, H_2_-rich saline protected the retina against glutamate-induced excitotoxic injury in guinea pigs^28^. In the anterior eye segment, H_2_ prevented corneal endothelial damage in phacoemulsification cataract surgery^29^ and suppressed oxidative stress in the cornea of experimental animals evoked by corneal alkali burns, using a lower^30^ as well as higher^7^ concentration of alkali. As already mentioned, in this study H_2_ prevented or highly reduced the oxidative damage of UVB irradiated corneas, leading to the restoration of transparency. The corneas healed without neovascularization and scar formation. This was in contrast to irradiated untreated or PBS treated corneas, which were untransparent and vascularized.

The article "Therapeutic effect of molecular hydrogen in corneal UVB-induced oxidative stress and corneal photodamage" was retracted in 2021. Reason: duplicated images.

## Results

In our study, apart from the group of rabbits with UVB irradiated corneas treated with H_2_ solution or with PBS (H_2_ free), there was the group of rabbits, which were left without any treatment during and after UVB irradiation. As the immunohistochemical, biochemical and macroscopical results of irradiated untreated corneas did not significantly differ from the results obtained with irradiated corneas treated with PBS (H_2_ free), we did not show the results of the irradiated untreated group.

### The H_2_ solution treatment of UVB irradiated corneas prevented the development of the antioxidant/prooxidant and protease/antiprotease imbalance in the corneal epithelium

The first irradiation of the cornea with UVB rays already caused the imbalance between antioxidant and prooxidant enzymes in the corneal epithelium in untreated or buffer treated corneas. The expression of antioxidant enzymes (superoxide dismutase, SOD, glutathione peroxidase, GPX, catalase, CAT) (shown with SOD were decreased, whereas the expressions of prooxidant enzymes (oxidases that generate ROS) (xanthine oxidase, XOX, D-amino acid oxidase, DAAO) (shown with the expression of XOX). remained unchanged or even increased. This was followed by the protease/antiprotease imbalance in the corneal epithelium. The expressions of MMPs (MMP2, MMP9) (shown with MMP9) were increased, while the expressions of TIMPs (TIMP2, TIMP4) (shown with TIMP2) were decreased. When the corneas were treated with H_2_ solution during irradiation, the antioxidant/prooxidant balance as well the protease/antiprotease balance, remained unchanged in the corneal epithelium compared to the control corneas. The expression of individual antioxidant and prooxidant enzymes, as well as MMPs and TIMPs, were similar to those in the control epithelium (images are shown in supplementary data). Here we show the expression of genes for MMP2 and MMP9 in irradiated corneas treated with H_2_, irradiated corneas treated with buffer (free of H_2_) and control corneas quantified by real-time PCR (day 16). The treatment of irradiated corneas with H_2_ solution significantly decreased the expression of metalloproteinases compared to irradiated buffer treated corneas (Fig. 1D,E).

**Figure 1:** H_2_ solution treatment prevents enzymatic changes in the corneal epithelium. At the end of experiment (day 16) the expression of genes for K3 and K12 quantified by real-time PCR showed that the treatment of irradiated corneas with H_2_ solution significantly increased the expression of K3 and K12 (**A**,**B**). The values with astericks are significantly different (*p < 0.05, ***p < 0.001) from buffer treated irradiated corneas. The expression of genes for MMP2 and MMP9 quantified by real-time PCR showed that the treatment of H_2_ significantly decreased the expression of MMP2 and MMP9 in irradiated corneas (**D**,**E**). The values with astericks are significantly different (**p < 0.01) from buffer treated irradiated corneas. At the same time inerval (day 16) the irradiated corneas treated with H_2_ show high expression of K3/K12 detected immunohistochemically (**C**). Scale bars: 50 µm.

The article "Therapeutic effect of molecular hydrogen in corneal UVB-induced oxidative stress and corneal photodamage" was retracted in 2021. Reason: duplicated images.

### The treatment of UVB irradiated corneas with H_2_ solution increased the expression of keratin 3 (K3) and keratin 12 (K12) in the corneal epithelium

The expression of genes for K3 and K12 in control (healthy), irradiated PBS treated and irradiated corneas treated with H_2_ solution quantified by real-time PCR, showed that the treatment of irradiated corneas with H_2_ solution significantly increased the expression of K3 and K12 (day 16) (Fig. 1A,B). The immunohistochemical expression of K3/K12 was high in irradiated corneas treated with H_2_ solution (compared with control corneas), whereas the expressions were low in irradiated corneas treated with PBS, where only flat epithelium was present and some corneas were without epithelium (Fig. 1C).

### The influence of H_2_ solution treatment of UVB irradiated corneas on the expression of intrleukin-1β (IL-1β), transforming growth factor-β (TGF-β), malondialdehyde (MDA) and nitrotyrosine (NT) in corneas

The expression of IL-1β, TGF-β (Fig. 2A,B), MDA and NT (Fig. 2C,D) detected immunohistochemically and by real-time PCR were high in irradiated corneas treated with PBS, whereas they were low or absent in irradiated corneas treated with H_2_ solution (day 16), similarly as in control corneas.

**Figure 2:** H_2_ solution treatment reduced corneal inflammation and oxidative stress. H_2_ solution dropped on the corneal surface during irradiation and then during corneal healing decreased the induction of pro-inflammatory cytokines in corneas (shown with IL-1β and TGF-β) (**A**,**B**) and prevented the immunohistochemical expression of MDA and NT in irradiated corneas (**C**,**D**). Scale bars: 50 µm. The values with astericks are significantly different (*p < 0.05, **p < 0.01, ***p < 0.001) from buffer treated irradiated corneas.

### The H_2_ solution treatment of UVB irradiated corneas with reduced apoptosis of corneal cells and protected corneas against neovascularization and scar formation

The number of apoptotic cells in irradiated corneas treated with H_2_ solution was significantly reduced compared to buffer treated irradiated corneas (Fig. 3A,C). The expression of vascular endothelial growth factor (VEGF) was also significantly reduced in irradiated corneas treated with H_2_ solution, whereas in buffer treated irradiated corneas, the expression was high (Fig. 3A,D). Representative photographs of healthy and irradiated eyes treated with H_2_ solution or PBS are shown in Fig. 4A, and the number of vessels in Fig. 4B. In comparison with the irradiated eyes treated with H_2_ solution, which remained transparent and without vessels until the end of the experiment (day 16), the irradiated corneas treated with buffer became opalescent early after the irradiation. At the end of the experiment (day 16) the corneas were vascularized and untransparent.

The article "Therapeutic effect of molecular hydrogen in corneal UVB-induced oxidative stress and corneal photodamage" was retracted in 2021. Reason: duplicated images.

**Figure 3:** Corneal apoptosis and neovascularization decreased after H_2_ solution treatment. H_2_ supresses apoptosis of corneal cells (arrow, showed with active caspase-3) (**A**,**C**) and reduced VEGF expression detected immunohistochemically **(A**) and VEGF gene expression quantified by real-time PCR (**D**). The values with astericks are significantly different (*P < 0.05, ***P < 0.001) from buffer treated irradiated corneas. Scale bars: 50 µm.

**Figure 4:** The renewal of corneal transparency after H_2_ solution treatment. Representative photographs of healthy and irradiated treated eyes. Corneal opalescency seen after the injury early disappeared after H_2_ treatment. Afterwards (from day 4 to day 16) the corneas were transparent. Corneal neovascularization and scar formation were prevented (**A**,**B**). In corneal neovascularization the values with astericks are significantly different (***P < 0.001) from buffer treated irradiated corneas (day 16).

### The H_2_ solution treatment of UVB irradiated cornea reduces the increase in central corneal thickness (central corneal thickness considered an index of corneal hydration)

Shortly after irradiation, in buffer treated corneas, the central corneal thickness increased more than twice (compared to levels before injury, day 0) in buffer treated irradiated corneas, it later decreased but, the values remained elevated until the end of the experiment (day 16). In H_2_ treated irradiated corneas the central corneal thickness was slightly increased after repeated irradiation, compared to levels before irradiation, and from day 10 the corneal thickness returned to the values before irradiation (day 0) (Fig. 5).

**Figure 5:** The effect of H_2_ solution treatment on central corneal thickness. Central corneal thickness (taken as an index of corneal hydration) was measured in the same rabbit before irradiation (day 0) and after the irradiation and treatment with H_2_ or buffer alone (free of H_2_). In the buffer treated irradiated corneas, the values were statistically different from the values before irradiation in all time intervals, until the end of experiment (day 16). In contrast, H_2_ solution treatment prevented the high increase in central corneal thickness and from day 10 the values were not significantly different from the values before irradiation (day 0). The values with astericks are significantly different (*p < 0.05, **p < 0.01, ***p < 0.001) from values before irradiation (day 0).

The article "Therapeutic effect of molecular hydrogen in corneal UVB-induced oxidative stress and corneal photodamage" was retracted in 2021. Reason: duplicated images.

The differences in corneal healing after buffer treatment or H_2_ solution treatment of UVB irradiated corneas are summarized in Fig. 6.

**Figure 6:** Schematic modul of H_2_ solution treatment vs. buffer treatment. Differences in the healing results of UVB irradiated corneas, treated with H_2_ solution and buffer (free of H_2_), are summarized. The substantial effect of H_2_ treatment consists in the suppression of oxidative stress evoked by UVB radiation.

## Discussion

Oxidative stress has been found to be implicated in the pathogenesis of various corneal injuries and diseases, such as corneal irradiation with UVB rays, corneal alkali burns, dry eye disease, keratoconus, Fuchs’ endothelial dystrophy and bullous keratopathy^7–9,30–33^. The expressions of MDA (a marker of lipid peroxidation) and NT (a marker of oxidative stress) were described in diseased corneas in the cells of individual corneal layers. He results of this paper show that the H_2_ solution dropped on the ocular surface during irradiation, and during healing, prevented or highly suppressed MDA and NT expressions in irradiated corneas. This was in contrast to untreated or buffer treated irradiated corneas where MDA and NT were present (Fig. 2C,D).

The eye, and particularly the anterior segment, are directly open to environmental influences such as UVB radiation which makes them susceptible to oxidative stress. The eye contains low molecular weight antioxidants such as ascorbic acid, glutathione and alphatocopherol), as well as high molecular weight antioxidant enzymes (CAT, SOD and GPX), which play a key role in protecting the eye against oxidative damage. SOD catalyzes the dismutation of superoxide to hydrogen peroxide and molecular oxygen. Therefore, this enzyme protects the ocular tissues against superoxide radicals. GPX, together with CAT, are very important scavengers of hydrogen peroxide. In the normal eye there exists a balance between prooxidants and antioxidants. The danger to the eye appears under various injuries or diseases, such as the irradiation of the eye with UVB rays, when the antioxidant/prooxidant balance is disturbed. Previous papers suggested the involvement of xanthine oxidoreductase/xanthine oxidase^3,4,34–36^ that generates ROS in the development of this imbalance^8,9^ and the appearance of oxidative stress. Oxidative stress stimulates the production of unstable and highly reactive oxygen and nitrogen related products, that are responsible for cellular damage. To combat the ubiquitous presence of ROS, ocular tissues have evolved diverse antioxidant defence systems, to prevent permanent and lasting ROS-mediated tissue damage. However, when prooxidants overwhelm the antioxidant defences, oxidative stress appears leading to the development of ocular pathologies^4,33,37^. For the insufficiency of antioxidants, therapeutic natural and nutraceutical anti oxidants were proposed for the treatment of eye diseases (e.g. Richer^38^). However, the use of such supplements might produce inconsistent results^16,39^. Ohsawa *et al*.^10^ proposed that H_2_ has potential as a novel effective antioxidant in preventive and therapeutic applications. H_2_ can be consumed in the human body by various ways, including inhaling H_2_, drinking hydrogen water (H_2_-dissolved water), taking a hydrogen bath, injecting H_2_ dissolved saline, dropping H_2_ solution onto the eye, and increasing the production of intestinal H_2_ by bacteria^16,21,40^. According to these authors, H_2_ has a number of advantages as a mild but effective antioxidant: H_2_ rapidly diffuses into tissues and cells, and it is not mild enough either to disturb metabolic redox reactions, or to affect ROS that function in cell signaling. H_2_ is an inert gas and only the strong oxidants, for example, hydroxyl radicals and NT, are able to oxidize them. The antioxidant effects of H_2_ was shown in this study. After the treatment of UVB irradiated corneas with H_2_ solution, the antioxidant/prooxidant balance and protease/antiprotease balance, present in the healthy corneal epithelium, were not disturbed, whereas in the irradiated epithelium treated with PBS free of H_2_ the antioxidant/prooxidant and protease/antiprotease imbalances developer, contributing to oxidative and nitrosative stress. This leads to the increased expression of MMPs (Fig. 1A,B), the decreased expression of TIMPs and to the induction of proinflammatory cytokines. (Figs 1 and 2). This was found in our study in UVB irradiated corneas treated with PBS (free of H_2_). The local release of proinflammatory cytokines and proteases by cells in UVB irradiated corneas, is highly responsible for UVB-mediated corneal inflammation and cell death^8,9^. In UVB irradiated corneas, the expression of nitric oxide synthases that generated nitric oxide were increased and elevated levels of nitric oxide were found in the aqueous humor^8^. NT, a toxic reaction product of nitric oxide and superoxide, which serves as an important marker of free radical damage, appeared in the cornea. Elevated NT staining was also found in this study in buffer treated irradiated corneas and H_2_ application prevented or highly decreased NT expressions. In addition to antioxidant functions, the anti-inflammatory and anti-apoptotic properties of H_2_ were shown in the present study. H_2_ downregulated proinflammatory cytokine and prevented the activation of caspase-3, which reduced apoptosis (Figs 2 and 3). This corresponds with the results obtained previously in various diseased organs following H_2_ therapy^31^. According to Slezak *et al*.^41^ H_2_ can also induce cytoprotection, probably due to the potentiation of antioxidant enzymes, such as SOD and CAT. H_2_ also regulates various signal pathways and the expression of many genes^16,21,40^.

The article "Therapeutic effect of molecular hydrogen in corneal UVB-induced oxidative stress and corneal photodamage" was retracted in 2021. Reason: duplicated images.

The corneas treated with H_2_ during irradiation, healed with the restoration of transparency without neovascularization and scar formation. This was in contrast to PBS (free of H_2_) treated corneas, which were untransparent and vascularized. According to Kubota *et al*.,^30^ inflammation is the trigger of angiogenesis after injury. However, ROS formation by alkali injury, or irradiation of the cornea with UVB rays, precedes the inflammatory response. For this reason, the H_2_ therapy is very effective. We can show in our study that intervention with H_2_ during UVB irradiation and healing, prevented or highly suppressed corneal neovascularization. The expression of MMPs and VEGF, all implicated in the development of corneal neovascularization, were decreased after H_2_ treatment (Figs 1, 3 and 4).

A healthy, transparent cornea is essential for good vision. The transparency of the corneal stroma is critically dependent on the levels of corneal hydration. Transparency of the cornea is a consequence of the detailed ultrastructure of the tissue and has been attributed to the narrow uniform diameter collagen fibrils, and to the regularity of their lateral packing. If the cornea swells, light scattering appears. According to the Meek *et al*.^42^, this scattering has been ascribed to the disruption caused to the arrangements of collagen fibres. Changes in the refractive index of the extracellular materiál, make only a small contribution to the increase in light scattering when the cornea swells. Altered corneal transparency, due to increased corneal hydration, was already described by Zucker^43^ and in UVB irradiated corneas by Cejkova *et al*.^8,9^. We report similar findings in this study in corneas treated with PBS free of H_2_. Corneal hydration was largely increased after the irradiation and remained elevated until the end of the experiment. In contrast, after H_2_ application during UVB irradiation, the increase in corneal hydration and decrease of transparency were significantly less pronounced during the whole experiment and it reached levels before irradiation at the end of the experiment (Fig. 5). Corneal hydration was evaluated by the measuring of the central corneal thickness, taken as an index of corneal hydration using an ultrasonic pachymeter.

The article "Therapeutic effect of molecular hydrogen in corneal UVB-induced oxidative stress and corneal photodamage" was retracted in 2021. Reason: duplicated images.

To the best of our knowledge, this study is the first to descibe the protective effect of H_2_ against the damaging effect of ROS, induced by UVB irradiation of the rabbit cornea. We have shown that H_2_ highly suppressed oxidative stress in the UVB irradiated cornea. The development of the antioxidant/prooxidant and protease/antiprotease imbalance was prevented or reduced in the irradiated corneal epithelium, leading to the decrease of corneal inflammation and beneficial corneal healing. It can be concluded that H_2_ proved to be a potent nontoxic antioxidant, suitable for therapeutic use in the prevention of ocular photodamage.

## Material and Methods

### Preparation of H_2_ solution in PBS

In our experiments, original Dr. Hidemitsu Hayashi’s Hydrogen Rich Water Stick and original Dr. Hayashi Glass Bottle (The Hydrogen Rich Water Group LLC Lawrence, Kansas, USA) were used. The special glass bottle was filled with the PBS and the hydrogen stick was immersed into the bottle. Then the bottle was tightly closed without the dead volume. The bottle was shaken for 15 sec and left to stand for 45 min. Afterwards the stick was taken out of the bottle. The small amount of missing solution was refilled with PBS and the bottle tightly closed.

### Measuring H_2_ concentration in PBS solution

For the measuring of the concentration of the dissolved molecular hydrogen in PBS (pH 7.2 continually checked by pH meter) the Trustlex ENH-1000 (TRUSTLEX, Kyoto, Japan) was used as the primary measuring device (see Cejka *et al*.^7^ in detail). In brief: The Trustlex ENH-1000 is an original Japanese made device for measuring dissolved hydrogen and it displays the dissolved hydrogen by means of hydrogen reduction method in ppm units (wt of H_2_/vol of solution). The device is calibrated directly in ppm (the readings are in ppm).

As a control method for the measuring of molecular hydrogen concentration in PBS buffer, the Unisense H_2_ Microsensor was employed. This microsensor is the Clark-type sensor measuring hydrogen partial pressure. The resulting sensor signal is in the pA current range. This signal is measured by the Unisense Microsensor Multimeter. The Multimeter readings can be transferred (according to the manual of the Multimeter) to the concentrations of the dissolved molecular hydrogen in PBS in mmol/L. The results obtained using both measuring methods differed in 15% of absolute values maximally.

For our experiments, the solution was stored in glass syringes equipped with stop cups. Attention was paid to the fact that no dead volume was present in the syringes. According to Ohta^16^, H_2_ can be dissolved in water up to 1.6 ppm, wt/vol (0.8 mM) under atmospheric pressure. In our study, the H_2_ concentration measured immediately after preparing the solution was 0.57 ± 0.9 ppm (wt/vol).

The article "Therapeutic effect of molecular hydrogen in corneal UVB-induced oxidative stress and corneal photodamage" was retracted in 2021. Reason: duplicated images.

### Animals

Adult, female New Zealand white rabbits (2.5–3.0 kg) obtained from Velaz Ltd. (Prague, Czech Republic, http://www.velaz.cz) were used in the experiments. The investigation was conducted according to the ARVO Statement for the Use of Animals in Ophthalmic and Vision Research and was approved by the Ethics Committee of the Institute of Experimental Medicine, Academy of Sciences of the Czech Republic, in Prague. Rabbits were anesthetized by an i.m. injection of Rometar (Xylazinum hydrochloricum, Spofa, Prague, CR, 2%, 0.2 ml/1 kg body weight) and Narkamon (Ketaminum hydrochloricum, Spofa, 5%, 1 ml/1 kg body weight). The corneas of anesthetized rabbits were irradiated with a daily dose of 1.0 J/cm^2^ for four days.

### Irradiation of the corneas with a UVB dose of 1.0 J/cm^2^

The open right eyes of anesthetized rabbits were irradiated with a UVB lamp (Bioblock Scientific, Illkirch Cedex, France; 312 nm wavelength, 6 W) at a daily dose of 1.0 J/cm^2^ for four days (six rabbits in the group, the whole experiment repeated twice). The animals were divided into three groups, in the first group the irradiated right eyes were treated with H_2_ solution, in the second group of animals, the right eyes were treated with buffer (free of H_2_) and in the third group the animals were left untreated. The dropping of 10 drops of H_2_ solution or buffer (one drop approximately 30 µl on the ocular surface, after each irradiation was performed and then the dropping of eyes was repeated three times daily (three times ten drops) until the end of the experiment (day 16). For UVB irradiation, the UVB lamp was positioned at a distance of 0.03 m for 5 minutes, 30 s (a dose of 1.0 J/cm^2^, intensity 3 mW/cm^2^). Only the corneas were irradiated; the rest of the eye surface was protected from the UV radiation. For irradiation, a UV lamp stand with a precisely determined distance between the lamp and the eyes was employed. The plane of the lamp was parallel to the tangential plane of the eye (at a right angle to the optical axis of the eye). The dose and intensity of irradiation were measured with the UVB sensor, connected to the radiometer (both instruments manufactured by Cole-Parmer Inc., Vernon Hills, Illinois, USA. The UVC sensor (Cole-Parmer Inc.) was employed to detect any potential emission of UVC rays. There was no emission of UVC detected. The animals of the three groups were sacrificed on day 16. The corneas of irradiated eyes were employed for immunohistochemical and biochemical investigation. The corneas of normal (healthy) rabbits served as controls.

The article "Therapeutic effect of molecular hydrogen in corneal UVB-induced oxidative stress and corneal photodamage" was retracted in 2021. Reason: duplicated images.

### Immunohistochemical examinations

After sacrificing the animals, the eyes were enucleated and the anterior eye segments dissected out and quenched in light petroleum chilled with an acetone-dry ice mixture. Sections were cut on a cryostat and transferred to glass slides. Subsequently, the cryostat sections were fixed in acetone at 4 °C for 5 min. For the immunohistochemical detection of K3/K12, IL-1β, XOX, DAAO, SOD, GPX, CAT, NT, MDA, VEGF, MMP 9, MMP 2, TIMP 2, TIMP 4 and active caspase-3, the following primary antibodies were used: mouse monoclonal anti-XOX Ab-2 (NeoMarkers, Fremont, California, USA), sheep polyclonal anti-DAAO (Abcam, Cambridge, United Kingdom), mouse monoclonal anti-SOD, sheep polyclonal anti-CAT, sheep polyclonal anti-GPX (Biogenesis, Poole, United Kindom), goat polyclonal anti-MMP9, goat polyclonal anti-MMP2 (Santa Cruz Biotechnology, Santa Cruz, California, USA), polyclonal goat anti-TIMP2 and polyclonal goat anti-TIMP4 (Santa Cruz Biotechnology), mouse monoclonal anti-IL-6 (Abcam), mouse monoclonal anti-VEGF (Abcam). anti-K3/12 (Abcam), monoclonal mouse anti-NT (Abcam), polyclonal goat anti-MDA (US Biological, Swampscott, Massachusetts, USA). The binding of the primary antibodies was demonstrated using the HRP/DAB Ultra Vision detection system (Thermo Scientific, Fremont, California, USA) following the instructions of the manufacturer: hydrogen peroxide block (15 min), ultra V block (5 min), primary antibody incubation (60 min), biotinylated goat anti-mouse IgG (Lab Vision, Fremont, California, USA), or donkey anti-goat IgG (Santa Cruz Biotechnology) secondary antibody incubation (10 min) and peroxidase-labeled streptavidin incubation (10 min). Visualization was performed using a freshly prepared DAB substrate-chromogen solution. Cryostat sections in which the primary antibodies were omitted from the incubation media served as negative controls. Sections were counterstained with Mayer’s hematoxylin. Negative controls included the omission of the primary antibody. Some samples were counterstained with Mayers’ hematoxylin (Sigma-Aldrich, St. Louis, Missouri, USA). After the staining procedure, the samples were immediately examined using an Orthoplan Leitz light microscope equipped with a Leica DC 500 digital camera.

The counting of cells positive for active caspase-3, NT and MDA in corneas, was performed by an examiner without prior knowledge of the experimental procedure. Three randomly chosen fields of corneal sections (of the same field size and the same microscope magnification), from six corneas of each experimental animal group were used. For each cornea the mean value from the three fields was counted. For the morphological evaluation of corneas, haematoxylin-eosin staining of post-fixed cryostat sections was employed.

The article "Therapeutic effect of molecular hydrogen in corneal UVB-induced oxidative stress and corneal photodamage" was retracted in 2021. Reason: duplicated images.

### The determination of the corneal thickness

Changes of corneal optical properties after the injury and during healing were evaluated by measuring the central corneal thickness (taken as an index of corneal hydration) (see Cejka *et al*.,^7^ in detail). Briefly: The central corneal thickness was measured in anesthetized animals using an ultrasonic pachymeter SP-100 (Tomey Corporation, Nagoya, Japan) in the corneal center. The corneal thickness was measured in the same corneas before irradiation (corneas of healthy eyes) and two, five, ten and sixteen days after the injury (all experimental groups). Each cornea was measured four times and the mean value of the thickness (in µm) was computed.

### The detection of gene expression by real-time PCR

The expression of genes for K3, K12, IL-1β, VEGF, MMP2 and MMP9 in control and treated corneas was determined by quantitative real-time polymerase chain reaction (PCR). Corneas were excised using Vannas scissors, transferred into Eppendorf tubes, and immediately frozen. The frozen corneal tissue was then homogenized and added in 500 μL of TRI Reagent (Molecular Research Center, Cincinnati, OH) for the RNA isolation. Total RNA was extracted using TRI Reagent according to the manufacturer’s instructions. One μg of total RNA was treated using deoxyribonuclease I (Promega, Madison, Wisconsin, USA) and subsequently used for reverse transcription. The first-strand cDNA was synthesized using random primers (Promega) in a total reaction volume of 25 μL, using M-MLV Reverse Transcriptase (Promega). Quantitative real-time PCR was performed in a StepOnePlus real-time PCR system (Applied Biosystems, Foster City, California, USA). The relative quantification model with efficiency correction was applied to calculate the expression of the target gene in comparison with GAPDH used as the housekeeping gene. The following primers were used for amplification: GAPDH: 5′-CCCAACGTGTCTGTCGTG (sense), 5′-CCGACCCAGACGTACAGC (antisense), VEGF: 5′-CGAGACCTTGGTGGACATCT (sense), 5′-ATCTGCATGGTGACGTTGAA (antisense), K3: 5′′-GAACAAGGTCCTGGAGACCA (sense), 5′-TTGAAGTCCTCCACCAGGTC (antisense); K12: 5′′-AGGAGGTGGTGAATGGTGAG (sense), 5′-GTTGTTTCCCAGGAGCAAAA (antisense). IL-1β 5′-CTGCGGCAGAAAGCAGTT (sense), 5′-GAAAGTTCTCAGGCCGTCAT (antisense), MMP2, 5ˇ-GTCTACTCGCTGGACATCGG (sense), 5′-GTGTATTCAGCCAGCACCCT (antisense), MMP9: 5′-AAGTTGGAAGTGGTGGCACA (sense), 5′-CGTCTTCCTGGGCAAAGAGT (antisense). The PCR parameters included denaturation at 95 °C for 3 min, then 40 cycles at 95 °C for 20 s, annealing at 60 °C for 30 s, and elongation at 72 °C for 30 s. Fluorescence data was collected at each cycle after an elongation step at 80 °C for 5 s and was analyzed on the StepOne Software, version 2.2.2 (Applied Biosystems). Each individual experiment was done in triplicate. In figure legends each bar represents the mean ± SD from 6 individual corneas. In Fig. 1 the value of control corneas for K3 and K12 is taken as 100% corresponding to the values of relative gene expression 18800 for K3 and 1750 for K12. In Fig. 2 the value of control corneas for IL-1β is taken as 100% corresponding to the value of relative gene expression 120. In Fig. 5 the value of control corneas for VEGF is taken as 100% corresponding to the value of relative gene expression 440.

The article "Therapeutic effect of molecular hydrogen in corneal UVB-induced oxidative stress and corneal photodamage" was retracted in 2021. Reason: duplicated images.

### Statistical analysis

The analysis of data showed normal distribution and the results are expressed as mean ± SD. Comparisons between two groups were made by Student *t*-test, and multiple comparisons were analyzed by ANOVA and post hoc test. A value of *p* < 0.05 was considered statistically significant. For corneal thickness, paired t-test was employed.

## Electronic supplementary material

Supplementary Information
